The article "Investigation of Estrogen Receptor (ESR1) for Breast Cancer from Traditional Chinese Medicine" was published in 2014. Journal: Biomed Res Int.

# Investigation of Estrogen Receptor (ESR1) for Breast Cancer from Traditional Chinese Medicine

**DOI:** 10.1155/2014/321486

**Published:** 2014-06-26

**Authors:** Tzu-Chieh Hung, Wen-Yuan Lee, Kuen-Bao Chen, Yueh-Chiu Chan, Calvin Yu-Chian Chen

**Affiliations:** ^1^Department of Biomedical Informatics, Asia University, Taichung 41354, Taiwan; ^2^School of Medicine, College of Medicine, China Medical University, Taichung 40402, Taiwan; ^3^Department of Neurosurgery, China Medical University Hospital, No. 2 Yude Road, North District, Taichung 40447, Taiwan; ^4^Department of Anesthesiology, China Medical University Hospital, Taichung 40447, Taiwan; ^5^Research Center for Chinese Medicine & Acupuncture, China Medical University, Taichung 40402, Taiwan; ^6^Human Genetic Center, Department of Medical Research, China Medical University Hospital, Taichung 40447, Taiwan

## Abstract

Recently, an important topic of breast cancer had been published in 2013. In this report, estrogen receptor (ESR1) had defined the relation of hormone-cause breast cancer. The screening of traditional Chinese medicine (TCM) database has found the molecular compounds by simulating molecular docking and molecular dynamics to regulate ESR1. S-Allylmercaptocysteine and 5-hydroxy-L-tryptophan are selected according to the highest docking score than that of other TCM compounds and Raloxifene (control). The simulation from molecular dynamics is helpful in analyzing and detecting the protein-ligand interactions. After a comparing the control and the Apo form, then based on the docking poses, hydrophobic interactions, hydrogen bond and structure variations, this research postulates that S-allylmercaptocysteine may be more appropriate than other compounds for protein-ligand interaction.

## 1. Introduction

There is an important topic of breast cancer that had been published in 2013. In this report, the estrogen receptor (ESR1) had defined the relation of breast cancer [1].

The breast cancer is a common cause of death in women and may originate either hormonally [2–5] from hereditary factors [6–9] and some other reasons [10]. Although there are lots of methods to find breast cancer based on accurate prediction, the surgery treatment causes patient low emotion from losing breast. Thus the prevention and treatment early medicinal treatment is widely accepted.

The ESR1 is a ligand-activated transcription factor that mediates the biological effects of the steroid hormone estrogen [11, 12]. From the inhibition of ESR1, the hormone would be regulated then decreased the risk for hormone breast cancer.

The Raloxifene is an FDA approval drug for reduction in the risk of breast cancer (http://www.cancer.gov/cancertopics/druginfo/fda-raloxifene-hydrochloride). The reference [13] had reported that the Raloxifene could target ESR1. For the above reason, the Raloxifene was chosen as the control for this investigation.

The article "Investigation of Estrogen Receptor (ESR1) for Breast Cancer from Traditional Chinese Medicine" was published in 2014. Journal: Biomed Res Int.

The computer-aided drug design (CADD) is an* in silico* simulation technique used in the screening of compounds based on the structure and biological activity. The CADD has the advantages of both greater speed and lower cost than the traditional drug design. The two major application areas of CADD are structure-based drug design and ligand-based drug design [14–17]. CADD is used to investigate drug design application centered on structure-based drug design and molecular dynamics.

The personalized medicine and biomedicine [18] are a novel department knowledge which could analyze the mutation [19], and the cause for special disease [20]. The traditional Chinese medicine (TCM) is defined a model case in this department. TCM has an important diagnosis culture in Asia, especially in China, Taiwan, Korea, and Japan. The TCM Database@Taiwan (http://tcm.cmu.edu.tw/) [21] is the largest traditional Chinese medicine database in the world. Since it was established in 2011, there have been successful discoveries of novel lead compounds from the TCM Database@Taiwan application for cancer treatment [22–25], memory disease prevention [26], pain relief [15], and antivirals [27–31]. Today, the screening of TCM compounds is possible from the application system of the website [32] and the cloud computing platform [33].

In this research, we screen a candidate compound against breast cancer from the TCM Database@Taiwan. The computational techniques of docking screening are used to select ligands prior to applying molecular simulation by molecular dynamics (MD) to investigate the variations in protein-ligand interactions that may contribute to the evaluation of the effects on ESR1 inhibition.

## 2. Materials and Methods

### 2.1. Data Set

A total of 61,000 TCM compounds were downloaded from the TCM database (http://tcm.cmu.edu.tw/). The human ESR1 (PDB ID: 1GWQ) crystal structure was obtained from RCSB Protein Data Bank [1, 13]. The Accelrys Discovery Studio 2.5 (DS 2.5) was used as the molecular simulations platform.

### 2.2. Disorder Protein Detection

The disorder region in protein plays an important role in drug design; thus we take the sequence to predict the disorder region by the Database of Protein Disorder (DisProt: http://www.disprot.org/) [34]. The prediction decides the character of protein structure; then taking the comparison with the docking site could evaluate the efficacy of the drug during protein-ligand interaction.

### 2.3. Molecular Docking

The LigandFit module [35], a receptor-rigid docking algorithm program in Discovery Studio 2.5 (DS 2.5), was used for docking simulations of Raloxifene and TCM compounds to ESR1 in the CHARMm force field [36]. The docking site of ESR1 was designed on the basis of the research [1, 13]. Through docking simulation, the top two compounds with the highest docking scores of the TCM compounds were selected to make the analysis of the hydrophobic interactions by Ligplus [37, 38].

The article "Investigation of Estrogen Receptor (ESR1) for Breast Cancer from Traditional Chinese Medicine" was published in 2014. Journal: Biomed Res Int.

### 2.4. Molecular Dynamics Simulation

The ligands of candidate complex must be reprepared before applying MD simulation by using SwissParam (http://swissparam.ch/) [39] based on the reference force field [40] of GROMACS 4.5.5 [41]. The ESR1, with ligands, was placed in a simulation box in an appropriate buffer or other solution at a minimum distance of 1.2 Å from the complex. The solution for simulation was based on the TIP3P water model in which sodium and chloride ions were added to neutralize complex charges. Based on the Steepest Descent method for 5,000 steps to minimize the complex, the structure with the lowest energy was transferred to MD simulation. The electrostatic interactions were calculated on the basis of the particle-mesh Ewald (PME) method [42]. The calculation with each time step was 2 fs and the numbers of steps were 5,000,000 times then the total simulation time of MD was 10,000 ps. The equilibration under the 100 ps constant temperature (PER ensemble) was based on the Berendsen weak thermal coupling method. The protocols in Gromacs used the MD data to calculate the MD trajectories, RMSD, energy variations, and eigenvector after MD.

## 3. Results and Discussion

### 3.1. The Detection of Disorder Protein

The disorder protein is defined as unstructured protein which makes the compounds dock to protein and stabilize the complex with difficultly while the docking site is a disorder region. The cited references [17, 43] indicate that the disorder region may have lower side effect than the widespread domain. Thus the disorder region can be defined as a challenge for drug design. In the prediction, the residue with the disposition greater than 0.5 is defined as disorder region (Figure 1). In this result, all the important amino acids of ESR1 are less than the threshold; thus the disorder protein has a weaker effect on docking and simulation.

### 3.2. Molecular Docking

Ranking the result of molecular docking by docking score, the two top TCM compounds, and the control, were selected (Table 1). These TCM compounds are S-allylmercaptocysteine and 5-hydroxy-L-tryptophan, extract from the TCM herbs* Allium sativum* and* Mucuna pruriens*, respectively. The top compound, S-allylmercaptocysteine, is defined as an hepatoprotective and anticancer compound [44–54] and the herb* Allium sativum* has antimicrobial properties [55–57], ameliorates tamoxifen-induced liver injury [58], and prevents cancer [45, 59–62]. The second ranked herb,* Mucuna pruriens*, has been identified as being able to reduce oxidation and prevent Parkinson's disease [63, 64]. As mentioned above, the top-ranked compound could prevent or treat cancer. The second compound with antioxidation might ease symptoms of cancer. For the above reasons, we suggest that the selected compounds can have influence on ESR1.

The article "Investigation of Estrogen Receptor (ESR1) for Breast Cancer from Traditional Chinese Medicine" was published in 2014. Journal: Biomed Res Int.

The structure of control and the candidate compounds was selected after screening from the TCM database (Figure 2). The docking poses presents the ligands had interactions with different critical amino-acids in the protein.  Figure 3 indicates the selected compounds could target and interact with amino acids around docking site.

The hydrophobic interaction can be analyzed by Ligplus (Figure 4). This result shows that the amino acids Glu353, Leu391, Arg394, and Phe404 can interact with all ligands through hydrophobic interactions or hydrogen bonds, indicating that these amino acids might be important in ligand-protein binding situations.

### 3.3. Molecular Dynamics Simulation

The RMSD and energy variation of a complex during MD simulation were recorded (Figure 5). The total energy is in the range between −744 and −750∗10^3^ kJ/mol and tends to −748∗10^3^ kJ/mol. From this figure, if both the amplitude of complex RMSD and energy are less; then the simulation may become balanced. S-allylmercaptocysteine has larger variation than other ligands but the complex RMSD of S-allylmercaptocysteine is the lowest. From this situation, we suggest S-allylmercaptocysteine can still interact, and this interaction makes the complex more stable.

The RMSF focus on each residue was analyzed, and on the variation of the whole protein, including with the ligand interaction (Figure 6). In this result, it can be seen that the regions of protein-ligand interaction are similar.

The reference-identified eigenvector was used to represent the protein variation [65]. The first two eigenvectors were selected based on PCA (principal component analysis) calculation, and become the *X*- and *Y*-axes. The comparison with apo (unbound protein) could find protein variation of first main character of protein (Figure 7). The upper subunit in these figures are the first eigenvector diffusion between apo and complex. The following is a matrix established from first two eigenvectors. After the comparison, we find that complex with S-allylmercaptocysteine is similar to apo then different from other compounds. This situation may not mean an absence variation, but the position of variation might be smaller.

The article "Investigation of Estrogen Receptor (ESR1) for Breast Cancer from Traditional Chinese Medicine" was published in 2014. Journal: Biomed Res Int.

The clustering is a result of the division of data into several groups based on RMSD variation; thus data in the same group will have the similar structure (position and composition) (Figure 8). In this result, S-allylmercaptocysteine has the least group and the largest one is in last. This situation means the complex with S-allylmercaptocysteine will tend to balance quickly. The largest group of apo and 5-hydroxy-L-tryptophan is not in last and it might present this simulation for apo and 5-hydroxy-L-tryptophan is not enough. Thus S-allylmercaptocysteine and control, Raloxifene, might have better effect on ESR1.

After the structure variation discussion is based on eigenvector and clustering, we should take focus on the structure variation during protein-ligand interaction (Figures 9 to 11). In Figure 9(a), there is high percentage (100%) of H bond occupancy in Glu353 which indicates that Glu353 may have a function in the inhibition of ESR1 from Raloxifene interaction.  Figure 9(b) shows the variation between MD 0 ns and 10 ns which present the position and composition variation as control drug inhibit ESR1. As the variation of apo between 0 ns and 10 ns is smaller position variation, the variation of control might become a sample to detect the efficacy of compounds from the structure variation of simulation.

S-Allylmercaptocysteine has high H bond occupancy in both Glu353 and Arg394, with the variation in 2 and 5 being more variable than the control (Figure 10). This result might present that not only S-allylmercaptocysteine the efficacy as control, but also that the force might be stronger than control.

The 5-hydroxy-L-tryptophan complex interactions were recorded (Figure 11). Besides Glu353 and Arg394, Leu346 has been recorded in Figure 11(a). The structure variation of 5-hydroxy-L-tryptophan is more similar to S-allylmercaptocysteine than control. From this result, we suggest 5-hydroxy-L-tryptophan might also have the function for the inhibition of ESR1.

From these variations found, we suggest Glu353 might be important in inhibition and Arg394 might make the force stronger based on the H bond and structure variation.

The pathway definition is according to the calculation of caver 3.0 to determine the inter-path protein path during MD simulation [66]. The pathway could help to determine the ligand moving and the pole provided from protein after interaction (Figure 12). In these results, we could find a path through ESR1. We suggest the ligands inhibit ESR1 while the interaction is in the protein.

## 4. Conclusion

Based on the above discussion, we can find that the top two TCM compounds S-allylmercaptocysteine and 5-hydroxy-L-tryptophan can have effect on ESR1 against breast cancer. Glu353 might have important role in inhibition based on high H bond occupancy in MD. Finally, according to the discussion from docking, interaction, and variation, we suggest that S-allylmercaptocysteine might be the best compound to inhibit ESR1 against breast cancer, even better than the control.

The article "Investigation of Estrogen Receptor (ESR1) for Breast Cancer from Traditional Chinese Medicine" was published in 2014. Journal: Biomed Res Int.

## Figures and Tables

**Figure 1:** The disorder and binding site detection. The blue curve in the figure is the disorder disposition of each amino acid, and the red lines are the important amino acids for docking site designed.

**Figure 2:** The structure of control and candidate TCM compounds. (a) Raloxifene core, (b) S-allylmercaptocysteine, and (c) 5-hydroxy-L-tryptophan.

**Figure 3:** The docking poses of ligands. (a) The crystal structure of ESR1 and the docking site, (b) Raloxifene core, (c) S-allylmercaptocysteine, and (d) 5-hydroxy-L-tryptophan.

**Figure 4:** Ligplot illustrates the protein-ligand interactions. (a) Raloxifene core, (b) S-allylmercaptocysteine, and (c) 5-hydroxy-L-tryptophan. The deep red color of the hydrophobic interactions presents a high frequency in all ligand interactions.

**Figure 5:** Measures of the MD trajectories. (a) Complex RMSD, (b) ligand RMSD, and (c) the total energy.

**Figure 6:** The variation of RMSD focus on residue of protein. This figure compares the RMSF between apo and each ligand interaction.

**Figure 7:** The PCA-eigenvector between ligand and unbound protein. The projection to the first two PCA-eigenvectors as *X*-, *Y*-axes based on the backbone of ESR1. The comparison of eigenvector between apo (red) and ligand (blue). Each ligand is (a) Raloxifene core, (b) S-allylmercaptocysteine, and (c) 5-hydroxy-L-tryptophan.

**Figure 8:** The clustering for ESR1 in MD. (a) apo, (b) Raloxifene core, (c) S-allylmercaptocysteine, and (d) 5-hydroxy-L-tryptophan.

**Figure 9:** The variation of Raloxifene core and ESR1 complex in MD simulation. (a) H-bond variation, (b) structure variation. The (1)–(4) red color indicates the difference through MD.

**Figure 10:** The variation of S-allylmercaptocysteine and ESR1 complex in MD simulation. (a) H-bond variation, (b) structure variation. The (1)–(6) red color indicates the difference through MD.

**Figure 11:** The variation of 5-hydroxy-L-tryptophan and ESR1 complex in MD simulation. (a) H-bond variation, (b) structure variation. The (1)–(4) red color indicates the difference through MD.

**Figure 12:** The pathway of ESR1 for compounds. (a) Unbound protein, (b) Raloxifene core, (c) S-allylmercaptocysteine, and (d) 5-hydroxy-L-tryptophan.

The article "Investigation of Estrogen Receptor (ESR1) for Breast Cancer from Traditional Chinese Medicine" was published in 2014. Journal: Biomed Res Int.

**Table 1:** ESR1 basis PLP1, PLP2 and dock score sort screened top two from TCM database.

Name	Herb	-PLP1	-PLP2	Dock score
S-Allylmercaptocysteine	*Allium sativum *	49.96	49.61	182.706
5-Hydroxy-L-tryptophan	*Mucuna pruriens *	66.74	63.42	177.541
Raloxifene core∗		77.09	83.51	63.907

*Control.
